# Prevalence of Refractive Error in School Children in Suining City of Sichuan Province, China: A School-Based Cross-Sectional Study

This article has been retracted.

**DOI:** 10.1155/2022/4845713

**Published:** 2022-05-26

**Authors:** Linglin Liu, Heng Li, Zhijin Tang, Zaihong Huang, Xu Yang

**Affiliations:** Department of Ophthalmology, Central Hospital of Suining City, Suining, 629000 Sichuan Province, China

## Abstract

**Objective:**

To investigate the prevalence of refractive errors among school children in Suining City, Sichuan Province, and to provide a scientific basis for prevention and control of myopia.

**Methods:**

This was a school-based cross-sectional study. Children aged 6-15 years were selected from kindergartens, primary schools, and middle schools in the urban setting of Suining City. The children underwent ocular examination including measurement of uncorrected visual acuity (UCVA), visual acuity when wearing glasses, and noncycloplegic autorefractometry.

**Results:**

Of the 1200 eligible students, 1138 children (94.8%), 553 of them girls (47.4%), participated. The mean age was 10.64 ± 2.89 years. The prevalence of myopia, hyperopia, astigmatism, and emmetropia was 59.1% (95% confidence interval (CI): 57.6, 60.5), 5.0% (95% CI: 4.7, 6.1), 38.4% (95% CI: 55.5, 58.5), and 25% (95% CI: 23.7, 26.2), respectively. In univariate analysis, the prevalence of myopia was correlated with age, female gender, and learning stage. The prevalence of hyperopia and astigmatism was correlated with age and learning stage. The prevalence of mild myopia, moderate myopia, and high myopia in the 1138 students was 17.7%, 41.4%, and 3.3%, respectively. The prevalence of mild, moderate, and high myopia all increased with age and learning stage. The prevalence of myopia differed by gender. The mean spherical equivalents of the right and left eyes were −1.40 ± 1.99 diopters (D) and −1.29 ± 1.93 D, respectively, and the median values were -0.75 D and -0.6 D, respectively. The mean spherical equivalent increased with age, learning stage, and female gender.

**Conclusions:**

The most common type of refractive error was myopia which was associated with higher age, female gender, and higher learning stage. This study provides new data and recommendations for myopia-control in school-aged children in Sichuan province.

## 1. Introduction

Myopia is an increasingly serious public health problem around the world. It is estimated that 40% of the global population will suffer from myopia by 2030. By 2050, the prevalence of myopia will increase to 50%, and the number of people with high myopia will increase to about 900 million. The prevalence of myopia is about 56.9% in East Asia, which is significantly higher than that in other regions [1]. A 2013 study found that the prevalence of myopia in children 12 and 17 years old in East Asia were 52.5% and 59.1%, respectively, and that was significantly higher than in European teenagers (8.6% and 17.7%) [2]. A study in Singapore found that the prevalence of myopia was 63.4% in teenagers [3]. In Seoul, South Korea, the prevalence of myopia was 96.5% in males of an average age of 19 years, with about 10% to 20% of them suffering from high myopia [4, 5]. At present, the prevalence of myopia is high and growing rapidly among teenagers. According to the World Health Organization, there are 600 million myopic in China: it is estimated that 50% of them in primary school and 80% of them in junior and senior high school. In 2016, a study in the Jinshui District of Zhengzhou City showed that the prevalence of myopia was 38.5% among teenagers [6]. In 2017, the prevalence of myopia was 42.8% among multiethnic teenagers in Linxia Prefecture [7]. In 2017, a study of 3002 teenagers in Baoshan District of Shanghai showed the prevalence of myopia was 45.27% [8]. The prevalence of myopia increased year-by-year in Han children aged 7–18 years from 2005 to 2014, with the prevalence of myopia of 47.5%, 55.1%, and 57.1% in 2005, 2010, and 2014, respectively [9]. A study in Shanghai showed that the prevalence of myopia increased from 77.6% (2007) to 83.0% (2012) in primary and junior high school students [10]. In 2018, a study in China reported that the prevalence of myopia in primary school and junior high school students was 20% or 30% [11] every year. Myopia, especially high myopia, can be associated with ocular complications such as cataract, glaucoma, retinopathy, and vitreal diseases, which can lead to blindness, and thus lower the visual ability and quality of life of myopic and decrease the economic development of society. At present, high rates of myopia in teenagers are mainly concentrated in the developed areas in southern and eastern China, such as Shanghai [10], Guangzhou [12], Shandong [13], and Beijing [14]. The prevalence of myopia varies greatly in different regions and nationalities [15]. However, epidemiological data regarding ametropia among teenagers in Sichuan Province is limited, so more studies on ametropia are needed. This paper reports the prevalence of ametropia and myopia among children in Suining City, which provides reference data for an epidemiological survey of ametropia among teenagers, and provides a scientific basis for the formulation of myopia-prevention and -control programs in Sichuan Province.

## 2. Methods

### 2.1. Survey Samples

According to data from the census of 2010, the total resident population of Suining City is 3,252,551, including 130,900 students in school. That includes 45,100 students in primary school (with an enrollment rate of 99.74%) and 30,500 students in junior middle school (with an enrollment rate of 99.94%). Therefore, our study population was representative of the local pediatric population. This study used a cross-sectional survey method with stratified cluster sampling. The sample size was calculated by estimating an age-specific prevalence of refractive errors of 33.5% with a 20% error rate and a 95% confidence interval (95% CI). Assuming a nonresponse rate of 10%, the cluster sample size was 120 for each age group, so we needed to enroll 1200 children ages 6 to 15 years old in the survey. One kindergarten, one primary school, and one junior high school were selected at random in the urban area. Then, two classes were selected from each grade. The normal refractive state in children less than 6 years old is hyperopia, and errors could have been introduced if the study had included such young children, according to the diagnostic criteria of this study, so the kindergarten cohort only included children 6 years of age and over. There were about 60 students in each class, and 1200 students in total, in the study.

### 2.2. Eye Examinations

Two ophthalmologists and two optometrists completed the ophthalmic examinations, and one experienced doctor managed and supervised the whole process. This study was approved by the medical ethics committee and approved by the school officials and by the students who were invited to this study and their parents before the ophthalmic examination.

The international standard “E” chart (National standard GB 11533-2011), at a viewing distance of 5 m, was used to determine the uncorrected visual acuity (UCVA) and visual acuity when wearing glasses (presenting visual acuity). The lowest line of the chart and the eyes of the children were aligned at approximately the same height. The examiners were trained in a consistent manner, and the students were told not to squint during the examination. For each student, the right eye was tested before the left eye. The children were asked to start reading on the first line of the chart and to continue reading with the next lines. The end point of the examination was the lowest line on which the child could correctly identify the direction of at least four characters. If the children could not correctly read the 20/100 line at a distance of 5 m, the test was repeated at a distance of 1 m. If, at that distance, the children could still not read enough characters, visual acuity was tested (in order) as counting fingers, hand motion, light perception, or no light perception. The identification time allotted for each visual aid was not to exceed 3 s. A UCVA ≥ 20/20 was considered normal. When checking UCVA, the children did not wear any glasses. When checking their vision as it is in daily life, the children wore their prescription glasses. If they normally wore hard or soft contact lens, the children were to take their contact lens out one-half hour before the UCVA test. In children who wore an orthokeratology lens or lenses, the UCVA was recorded as the visual acuity of wearing glasses. We recorded UCVA, presenting acuity, whether the student usually wore correction and, if so, the type (e.g., glasses or soft contact lenses).

Autorefractometry was also performed. The instrument was operated by a professional optometrist and calibrated with a simulated eye every day. Each eye was tested at least three times, and the average value was recorded. The difference between the maximum and minimum values of the measured spherical refractive error and cylindrical refractive error had to be less than 0.5 diopters (D); otherwise, the measurements were repeated. To assure the quality of the measurements of visual acuity and refractometry, the examiners were repeatedly checked for the accuracy of their results. Refraction measurements were conducted after the students removed their glasses. Students who wore corneal contact lens took them out 30 minutes before refractometry was performed. Students who wore an orthokeratology lens did not undergo refraction. There was no auto-refractometry performed with mydriasis. If the UCVA was <20/20, and spherical equivalent (SE) was ≤-0.50 D or >+0.50 D or the cylinder was ≥0.75 D, it was recommended that the student be examined at a regular medical institution.

### 2.3. Statistical Analysis

Statistical analysis was performed using a commercial statistical software package (SPSS for Windows, version 21.0, IBM-SPSS, Chicago, IL). Quantitative data is presented as mean ± standard deviation, while qualitative data is presented as prevalence. The prevalence rate was compared with *χ*^2^ tests. *T-*tests and Kruskal-Wallis tests were used to compare the means. The data is presented with 95% CIs. All *P* values were two-sided and were considered statistically significant when the value was less than 0.05. Bivariate correlation analysis was used to check for binocular correlation. If there was a significant correlation between the two eyes, data from the right eye was to be used for the statistics.

Classification of ametropia was based on the presence of UCVA < 5.0. Myopia was defined as a refractive error (SE) of ≤-0.50 D in one or both eyes. Mild myopia was defined as a refractive error of ≤-0.50 D to >-3.0 D in one or both eyes. Moderate myopia was defined as a refractive error of ≤−3.0 D to ≥-6.0 D in one or both eyes. High myopia was defined as a refractive error of<-6.0 D in one or both eyes. Emmetropia was consequently considered to be a refractive error of >-0.50 D and ≤+0.50 D in both eyes. Hyperopia was defined as a refractive error of >+0.50 D. Astigmatism was defined as a cylindrical refractive error ≥+0.75 D in either eye. SE of the refractive error was defined as the sum of the spherical refractive error plus one-half of the cylindrical refractive error.

## 3. Results

### 3.1. Demographic Data

Of the 1200 students who were eligible and invited to participate in the study, 1138 students actually participated (response rate 94.8%). Their demographic details are presented in Table 1. Among the study participants, 585 were boys (52.5%), and 553 were girls (47.4%). The mean age was 10.64 ± 2.89 years. 435 students (38.2%) in the study were from kindergarten and the lower grades of primary school (grades 1-3), 333 students (2) were from the higher grades of primary school (grades 4-6), and 370 students (32.5%) were from junior high school. The mean SE of the right and left eye were −1.41 ± 1.99 D (median: -0.75 D; range: -10.5 D to +5.5 D) and −1.29 ± 1.95 D (median: -0.625 D; range: -11.875 D to +6.0 D). There was a high correlation between the two eyes (*r* = 0.884), so the right eye data were used for analyses.

### 3.2. Classification of Ametropia

Shown in Figure 1 are the ametropia classifications of all of the students (classified into myopia, hyperopia, and astigmatism).

The prevalence of myopia across all students was 59.1% (95% CI: 57.6, 60.5). With increasing age, the prevalence of myopia increased from 23% (95% CI: 19.0, 27.05) in 6-year-old students to 87% (95% CI: 84.1, 90.0) in 15-year-old students. The prevalence of hyperopia was 5.0% (95% CI: 4.7, 6.1) overall. The prevalence of hyperopia increased from 1% (95% CI: 0.4, 1.6) in 6-year-old students to 2% (95% CI: 1.4, 2.6) in 15-year-old students. The overall prevalence of astigmatism was 38.4% (95% CI: 55.5, 58.5). The prevalence of astigmatism decreased from 46% (95% CI: 29.4, 62.6) in 6-year-old students to 29% (95% CI: 26.8, 31.17) in 10-year-old students. Then, it increased slightly to 36% (95% CI: 33.8, 38.3) in 15-year-old students. The overall prevalence of emmetropia was 25% (95% CI: 23.7, 26.2). With increasing age, the prevalence of emmetropia was 50% (95% CI: 47.0, 53.0) in 6-year-old students, decreased gradually to 5% in the 15-year-old students (95% CI: 3.1, 6.9).

In univariate analysis, the prevalence of myopia was significantly correlated with age, female gender, and grade (*P* < 0.001). The prevalence of hyperopia and astigmatism was significantly associated with age and grade (*P* < 0.001), but did not differ significantly (*χ*^2^ = 0.125/0.8) between boys and girls (*P* = 0.25/0.47). The incidence of emmetropia decreased with age (Tables 2, 3, and 4).

### 3.3. Classification and Prevalence of Myopia

As shown in Table 5, the prevalence of mild, moderate, and high myopia in the 1138 students were 17.7%, 41.4%, and 3.3%, respectively. This means that the majority of the students had moderate myopia.

The prevalence of mild, moderate, and high myopia increased with age (*χ*^2^ = 187.1, *P* < 0.001). The prevalence of mild myopia increased from 1.9% (6-year-olds) to 46% (15-year-olds), which increased significantly from 13.3% (12-year-olds) to 30.3% (13-year-olds). The prevalence of moderate myopia increased from % (6-year-olds) to 41.3% (15-year-olds), which increased slowly and stable with age. The prevalence of high myopia increased from 1.9% (6-year-olds) to 8.7% (15-year-olds), with significant increases from 1.8% to 4.2% in 11- to 12-year-olds and from 5.7% to 8.7% in 14- to 15-year-olds.

The prevalence of myopia differed by gender (*χ*^2^ = 4.4, *P* < 0.05). The prevalence of mild myopia and high myopia in boys (20.5% and 3.8%) were higher than in girls (14.6% and 2.7%). The prevalence of moderate myopia in girls (47.6%) was higher than in boys (35.6%).

The prevalence of mild and high myopia increased with the grade (*χ*^2^ = 191.4, *P* < 0.001). Mild myopia increased from 3.9% (kindergarten and lower grades of primary school) to 37.3% (junior high school). High myopia increased from 1.1% (kindergarten and lower grades of primary school) to 6.4% (junior middle school). The prevalence of moderate myopia increased slowly with the grade (33.1% to 46.7%).

As shown in Figures 2 and 3 and Table 6, the mean SE of the right and left eyes were −1.40 ± 1.99 D and −1.29 ± 1.93 D, respectively, and the median values were -0.75 D and -0.6 D, respectively. Taking the right eye as an example, the mean SE increased with age (*χ*^2^ = 43.0, *P* < 0.001; Kruskal-Wallis test), which was -1.25 D in 6-year-olds and -2.87 D in 15-year-olds. The mean SE of the right eyes of boys and girls were -1.49 ± 2.05 D and -1.31 ± 1.90 D (*t* = −1.5, *P* < 0.001), respectively, and the median value was -0.75 D in both genders. The mean SE across grade were significantly different (*χ*^2^ = 46.0, *P* < 0.001; Kruskal-Wallis test): the mean SE increased with grade, the mean SE were −0.49 ± 1.29 D, −1.20 ± 1.78 D, −2.65 ± 2.17 D, respectively, and the median values were -0.25 D, -0.75 D, and -2.25 D, respectively, in the kindergarten and lower grades of primary school, the higher grades of primary school, and the junior high school.

## 4. Discussion

The main purpose of this study was to investigate the prevalence of myopia among 6- to 15-year-old children in Suining City, Sichuan Province. The method included measurements of UCVA and presenting visual acuity and autorefractometry. Before the examinations were carried out, the children and their parents completed a standardized questionnaire to obtain demographic information, and information on the types of ametropia, whether the children wore glasses and, if so, the type of glasses worn. The data were statistically analyzed to provide epidemiological data on the prevalence of myopia and related factors among children, to aid the control or prevention of juvenile myopia in Sichuan Province.

This study analyzed the refractive errors all of the students, including hyperopia, astigmatism, and mainly, myopia. The prevalence rate of myopia for these 6- to 15-year-old students was 59.1%, which is higher than rates found among primary and secondary school students in some rural areas of Shandong Province and Yunnan Province (36.9% and 39.1%, respectively) [13, 16]. The likely reasons are: the students from Suining City have a heavier learning burden and pressure in these urban schools than students do in rural schools, so the time for near-vision use of the eyes is long, and the time for outdoor activities is short; with the rapid development of science and technology, and the economy, multimedia devices are used more for teaching in urban schools; and usage of electronic devices is higher in the better economic conditions in urban areas; because of the greater exposure to nature in a rural setting, the students in rural schools have more time for outdoor activity to relax their eyes. In addition, the results in Shandong and Yunnan came from 6 to 10 years ago; since that time, there has been an increased prevalence of myopia in teenagers, year by year. As early as 2007, Yang et al. [17] had confirmed that myopia is related to the urban living environment. In this study, we did not perform optometry after mydriasis, and there may have been some “pseudomyopia” caused by overboard with eye. The prevalence observed in the present study is lower than the prevalence of myopia among 7- to 18-year-olds in Beijing in 2014 (64.9%) and 6- to 15-year-olds in Tianjin in 2016 (71.1%) [14, 18]. This may be due to the larger sample in the Beijing study, the better economic conditions of students in Beijing and Tianjin, their more-intense learning tasks and/or the different criteria used for myopia diagnoses.

The prevalence of hyperopia in our study was 5.0% (11.0% in 6- to 8-year-olds, 2.8% in 9- to 12-year-olds, and 2.5% in 13- to 15-year-olds); the prevalence decreased significantly with age after age 9 years, which is consistent with the results of a meta-analysis in 2014: it reviewed 40 cross-sectional studies and summarized that the rates of hyperopia were 8.4% before 6 years of age, 2% to 3% in 9- to 14-year-olds and only 1% in 15-year-olds [19]. In 2013, Lan et al. reported that the prevalence of hyperopia in children who were 3 to 6 years old was 20%, and that the prevalence gradually decreased after age 6 [20]. The Anyang study found that the proportion of hyperopia decreased with age (from 30.9% to 2.8% in 7- to 14-year-old students, respectively) [21]. It is known that most children are hyperopic at birth and develop into emmetropia with the increase in the ocular axis and increasing age. The reason for the relatively low proportion of hyperopia in our study is the relatively small sample of young children (under 7 years old). In recent years, the onset age of children's emmetropia and myopia is earlier than before; therefore, the prevalence of hyperopia in Anyang 6 years ago was higher than that in our study. The sample of children less than 6 years old should be increased in future research.

The prevalence of astigmatism in this study (38.4%) is similar to the values reported in southern Taiwan (32.9%) [22], Hangzhou (32.7%) [23], and Shandong (36.6%) [13], but significantly higher than those in multiethnic countries (Asian children (8.29%), European children (18.1%), non-Hispanic white children (6.33%), and Tunisian children (6.67%) [24–26]), which suggests that the prevalence of astigmatism in children and teenagers may be related to racial differences. As early as 2007, some scholars explained it from the perspective of genes [27]. The eyelid of Asian people are thick, and the compression of the cornea affects its curvature, resulting in a high prevalence of astigmatism. Our study found that the prevalence of astigmatism was 44.5% in students aged 6 to 8 years old, decreased gradually to 33.3% in students aged 9 to 12 years old, and rebounded to 37.7% in students aged 13 to 15 years old. There was a slight change in the prevalence of astigmatism with the age, which was similar to the results of a 2015 study on children's refractive errors (NICER) [28] in Northern Ireland. At present, it is generally believed that astigmatism in children mainly consists of mild astigmatism, compound-myopic myopia-astigmatism, and against-the-rule astigmatism, and some studies [29, 30] report that astigmatism is not significantly related to age or gender. A study conducted in Australia [31] reported that astigmatism is related to age in adults. The prevalence of astigmatism in this study may not be abnormal, due to the small age span of the children or to the sample size. We will increase the sample size and/or increase the age range in later research.

This study investigated the classifications of mild myopia, moderate myopia, and high myopia. We found that students of different ages, genders, and learning stages mainly had middle myopia. The overall prevalence of myopia in girls (62.2%) was higher than that in boys (59.1%), which is consistent with a large number of studies [32–37]. Krause et al. [38] reported in 1982 that the differences in myopia between boys and girls are determined by genetic factors, dietary factors, puberty, and amount of close work. As girls reach puberty and final body height earlier than boys do, it leads to a rise in the prevalence of myopia. Xie et al. [39] found that the prevalence of myopia in girls was higher than in boys, and that there was a relationship between sex hormones and myopia. Therefore, girls should be encouraged to take part in outdoor activities, relax, and adjust, to improve their diet, and to reduce the prevalence of myopia. However, recent studies in Ireland [40] (on 6- to 15-year-old students), northern India [41] (on 5- to 15-year-old students), and Hong Kong [42] reported that the prevalence of myopia in boys was higher than in girls. As early as in 2003, Zadnik et al. [43] found that among children with an average age of 10 years, boys have a longer ocular axis, which may lead to a higher prevalence of myopia in boys than girls. This result needs to be confirmed through a large number of studies involving children from different races, different age groups, and different genders. The difference between this study and other studies is that the prevalence of high myopia in boys (3.8%) was higher than that in girls (2.7%), whereas multiple studies have shown that the prevalence of high myopia in girls is higher than that in boys [44–47]. A study [48] reported that the rs9307551 gene, which is related to high myopia, is highly related to the Han female population. The age range was 6 to 15 years in our study, compared with a large number of studies that reported high myopia rates in older youth (>16 years old); further investigation is needed.

We found that the prevalence of myopia and the average refractive error increased with age and learning stage. This result is consistent with research results in other studies [49–52]. At present, it is generally believed that there is a relationship between the diopter of myopia and axial length. The analysis of myopia in 7- to 14-year-old children in the Wenzhou area [53] showed that the prevalence of myopia, axial length, and anterior-chamber depth all increase with age, which is consistent with our study. The reason is that during the development of refractive state, the axial length of the eyeball increases to constantly maintain the focus of the macula. When close work is performed, the tension of the choroid and ciliary muscles limits the expansion of the equator of the eyeball and the eyeball extends toward the back. Biochemicals, such as atropine and dopamine, also lead to the lengthening of the ocular axis. Learning tasks and learning pressure increase with increased learning stage, as students need to acquire more knowledge through repeated reading and writing, so students spend a lot of time at work. Additionally, students regularly use a variety of electronic products, including educational software, game software, and social software, which leads to increase near-work time. The above points confirm that the prevalence and average diopter of myopia are related to the age and learning stage. Therefore, to reduce the prevalence of myopia, we advocate reducing students' learning burden, preventing the use of electronic devices, and adhering to eyecare exercises and other eyecare measures.

The strengths of our study are: the sample in this epidemiological survey is representative of the local pediatric population. It is estimated that 1200 students were eligible, and a sampling cross-sectional survey method was adopted in this study, with one kindergarten, one primary school, and one junior high school randomly selected from all schools in the main urban area, and two classes selected from each grade. The above points avoided errors in the results due to unscientific sampling.

There are also limitations in this study: all the survey participants were school students, so we missed including children with low vision, who are not in school, and the deaf-mute children who are in special schools; high myopia mainly occurs in older youth, but our subjects were all under the age of 16; therefore, the prevalence and gender differences for high myopia need further study, and finally, we did not perform optometry after mydriasis, and so there may have been some cases of “pseudomyopia.” Autorefractometry after mydriasis would be needed to address that last issue.

In conclusion, the main type of refractive error among 6- to 15-year-old children in Suining City of Sichuan Province was myopia, particularly moderate myopia. The results of this study provide a strong scientific summary of the developmental trends and the factors influencing myopia in school students in Sichuan Province, which is of great significance to the formulation of prevention and control programs. Prevention and control of myopia require the joint efforts of students, parents, and medical and educational institutions.

## Figures and Tables

**Figure 1:** Prevalence of refractive errors of myopia, hyperopia, astigmatism and emmetropia stratified by age.

**Figure 2:** Distribution of refractive errors (spherical equivalent) of the right eyes, stratified by age and gender.

**Figure 3:** Distribution of the refractive errors (spherical equivalent) of the right eyes, stratified by age and grade.

**Table 1:** Enrolled and tested population stratified by age, gender, and grade in this study.

	Number (%) of students enrolled	Number (%) of students tested	Percentage tested (number enrolled/number tested) (%)
Age (years)			
6	120 (10.0)	108 (9.5)	96.4
7	120 (10.0)	110 (7.9)	91.7
8	118 (9.80)	110 (7.9)	93.2
9	115 (9.6)	107 (9.4)	93.0
10	115 (9.6)	110 (7.9)	95.7
11	115 (9.6)	110 (7.9)	95.7
12	118 (9.8)	113 (9.9)	95.8
13	124 (10.3)	122 (10.7)	98.4
14	125 (10.4)	122 (10.8)	97.6
15	130 (10.8)	126 (11.1)	96.9
Gender			
Male	610 (50.8)	585 (51.4)	95.9
Female	590 (49.2)	553 (48.6)	93.7
Grade			
Kindergarten and lower grade of primary school	450 (37.5)	435 (38.2)	96.7
High grade of primary school	355 (29.6)	333 (29.3)	93.8
Junior middle school	395 (32.9)	370 (32.5)	93.7
All	1200 (100.0)	1138 (100.0)	94.8

**Table 2:** Prevalence of myopia by age, gender, and grade.

	All (*n*)	Myopic (%)	Nonmyopic (%)	*χ* ^2^	*P* value
Age (years)					
6-8	328	98 (29.9%)	230 (70.1%)	187.1	<0.001
9-11	327	197 (60.2%)	130 (39.8%)		
12-15	483	377 (78.1%)	106 (21.9%)		
Gender					
Male	585	328 (56.1%)	257 (43.9%)	4.4	<0.05
Female	553	344 (62.2%)	209 (37.8%)		
Grade					
Kindergarten and lower grade of primary school	435	161 (37.0%)	274 (63.0%)	191.4	<0.001
High grade of primary school	333	196 (59.0%)	137 (41.0%)		
Junior middle school	370	315 (85.1%)	55 (14.9%)		
All	1138	672 (59.1%)	466 (40.9%)		

**Table 3:** Prevalence of hyperopia by age, gender, and grade.

	All (*n*)	Hyperopia (%)	Nonhyperopia (%)	*χ* ^2^	*P* value
Age (years)					
6-8	328	36 (11.0%)	292 (89.0%)	34.5	<0.001
9-11	327	9 (2.8%)	318 (97.2%)		
12-15	483	12 (2.5%)	471 (97.5%)		
Gender					
Male	585	28 (4.8%)	557 (95.2%)	0.125	0.25
Female	553	29 (5.2%)	524 (94.8%)		
Grade					
Kindergarten and lower grade of primary school	435	40 (9.2%)	395 (90.8%)	28.8	<0.001
High grade of primary school	333	13 (3.9%)	320 (96.1%)		
Junior middle school	370	4 (1.1%)	366 (98.9%)		
All	1138	57 (5.0%)	1081 (95.0%)		

**Table 4:** Prevalence of astigmatism by age, gender, and grade.

	All (*n*)	Astigmatism (%)	Nonastigmatism (%)	*χ* ^2^	*P* value
Age (years)					
6-8	328	146 (44.5%)	182 (55.5%)	8.8	<0.05
9-11	327	109 (33.3%)	218 (66.7%)		
12-15	483	182 (37.7%)	301 (62.3%)		
Gender					
Male	585	232 (39.7%)	353 (60.3%)	0.8	0.47
Female	553	205 (37.0%)	348 (62.9%)		
Grade					
Kindergarten and lower grade of primary school	435	188 (43.2%)	247 (56.8%)	11.6	<0.05
High grade of primary school	333	104 (31.2%)	229 (68.8%)		
Junior middle school	370	145 (39.2%)	225 (60.8%)		
All	1138	437 (38.4%)	701 (61.6%)		

**Table 5:** Prevalence (%) (95% confidence interval) of mild myopia, moderate myopia, and high myopia stratified by age, gender, and grade.

		Mild myopia (%) (95% CI)	Moderate myopia (%) (95% CI)	High myopia (%) (95% CI)
Age (years)	Number	(−0.5 D ≤ SE < −3.0 D)	(−3.0 D ≤ SE ≤ −6.0 D)	SE > −6.0 D
6	108	2 (1.9) (0.6-4.4)	23 (21.3) (14.3-28.3)	2 (1.9) (0.6-4.4)
7	110	5 (4.5) (0.7-11.5)	28 (25.5) (17.4-33.6)	2 (1.9) (0.6-3.2)
8	110	4 (3.6) (1.9-5.3)	36 (32.7) (28.3-37.1)	1 (0.9) (0.1-0.18)
9	107	6 (5.6) (3.4-7.8)	57 (53.3) (48.5-58.0)	1 (0.9) (0.1-0.18)
10	110	13 (11.8) (8.8-14.8)	46 (41.8) (37.1-46.5)	0
11	110	16 (14.5) (11.2-17.8)	59 (53.6) (48.9-58.3)	2 (1.8) (0.6-3.1)
12	113	15 (13.3) (10.1-16.5)	47 (41.6) (37.0-46.2)	5 (4.2) (2.4-6.0)
13	122	37 (30.3) (26.2-34.4)	61 (50.0) (45.5-54.5)	6 (4.9) (3.1-6.8)
14	122	45 (36.9) (32.6-41.2)	62 (50.8) (46.3-55.3)	7 (5.7) (3.7-7.7)
15	126	58 (46.0) (41.6-50.4)	52 (41.3) (37.0-45.6)	11 (8.7) (6.2-11.2)
Gender				
Male	585	120 (20.5) (12.4-28.6)	208 (35.6) (33.7-37.5)	22 (3.8) (3.1-4.5)
Female	553	81 (14.6) (13.1-16.1)	263 (47.6) (45.5-50.0)	15 (2.7) (2.1-3.3)
Grade				
Kindergarten and lower grade of primary school	435	17 (3.9) (3.0-4.8)	144 (33.1) (30.9-35.2)	5 (1.1) (0.6-1.6)
High grade of primary school	333	44 (13.2) (11.4-15.0)	152 (45.6) (42.9-48.3)	8 (2.4) (1.6-3.2)
Junior middle school	375	140 (37.3) (34.9-39.7)	175 (46.7) (44.0-49.4)	24 (6.4) (5.2-7.6)
All	1138	201 (17.7) (16.6-18.8)	471 (41.4) (40.0-42.8)	37 (3.3) (2.8-3.8)

Abbreviations: 95% Cl: 95% confidence interval; SE: spherical equivalent; D: diopters.

**Table 6:** Refractive error (diopters) stratified by age, gender, and grade.

	Refractive error (diopters)				
	Mean ± standard deviation	Median (25%, 75%)	Minimum, maximum	*χ* ^2^/*t*	*P*
Age (years)					
6	−0.22 ± 1.05	-1.25 (-0.375, -0.25)	-6.75, +2.12	43.0	<0.001
7	−0.33 ± 1.43	-1.25 (-0.53, -0.375)	-7.75, +3.50		
8	−0.49 ± 1.27	-1.25 (-0.875, -0.125)	-6.75, +2.625		
9	−0.95 ± 1.30	-0.75 (-1.625, -1.30)	-4.62, +5.25		
10	−1.09 ± 1.54	-0.62 (-1.50, -0.125)	-8.00, +1.25		
11	−1.47 ± 1.71	-0.93 (-2.28, -0.25)	-6.75, +1.00		
12	−1.05 ± 2.03	-0.50 (-1.50, -0.125)	-7.50, +5.50		
13	−2.24 ± 2.13	-1.87 (-3.40, -0.625)	-10.00, +3.50		
14	−2.63 ± 2.00	-2.18 (-3.906, -1.125)	-9.25, +0.37		
15	−3.06 ± 2.32	-2.87 (-4.375, -1.375)	-10.5, 2.12		
Gender					
Male	−1.49 ± 2.05	-0.75 (-2.625, -1.25)	-10.00, +3.37	-1.5	<0.001
Female	−1.31 ± 1.90	-0.75 (-2.00, -0.125)	-10.50, +5.50		
Grade					
Kindergarten and lower grade of primary school	−0.49 ± 1.29	-0.25 (-0.875, 0.125)	-7.75, +5.25	46.0	<0.001
High grade of primary school	−1.20 ± 1.78	-0.75 (-1.75, -0.125)	-8.00, +5.50		
Junior middle school	−2.65 ± 2.17	-2.25 (-4.00, -0.875)	-10.50, +3.50		
All	−1.40 ± 1.98	-0.75 (-2.25, -.0125)	-10.50, +5.50		

## Data Availability

The data that support the findings of this study are available from the corresponding author upon reasonable request.
